# Lung Nodule Segmentation and Recognition Algorithm Based on Multiposition U-Net

**DOI:** 10.1155/2022/5112867

**Published:** 2022-03-23

**Authors:** Na Zhang, Jianping Lin, Bengang Hui, Bowei Qiao, Weibo Yang, Rongxin Shang, Xiaoping Wang, Jie Lei

**Affiliations:** ^1^Department of Thoracic Surgery, Tangdu Hospital, Air Force Military Medical University, Xi'an, China; ^2^Department of Dermatology, Tangdu Hospital, Air Force Military Medical University, Xi'an, China

## Abstract

Lung nodules are the main lesions of the lung, and conditions of the lung can be directly displayed through CT images. Due to the limited pixel number of lung nodules in the lung, doctors have the risk of missed detection and false detection in the detection process. In order to reduce doctors' work intensity and assist doctors to make accurate diagnosis, a lung nodule segmentation and recognition algorithm is proposed by simulating doctors' diagnosis process with computer intelligent methods. Firstly, the attention mechanism model is established to focus on the region of lung parenchyma. Then, a pyramid network of bidirectional enhancement features is established from multiple body positions to extract lung nodules. Finally, the morphological and imaging features of lung nodules are calculated, and then, the signs of lung nodules can be identified. The experiments show that the algorithm conforms to the doctor's diagnosis process, focuses the region of interest step by step, and achieves good results in lung nodule segmentation and recognition.

## 1. Introduction

With the global spread of new crown disease, more and more scholars focus on lung disease [1]. Among them, lung nodules are the main lesions of the lung. Malignant lung nodules can develop into lung cancer, which seriously threatens human health. Due to the small proportion of lung nodules in the lung, doctors might inevitably produce missed detection and false detection in the detection process. Therefore, through the research of artificial intelligence, scholars use intelligent algorithms to assist doctors in making accurate diagnosis. Specifically, it includes the following three aspects:

*Lung parenchyma segmentation*: Karthikeyan and Valliammai [2] proposed a multithreshold algorithm to extract lung parenchyma region. Wei et al. [3] constructed a 3D model to segment lung parenchyma. Mansoor et al. [4] established a model to segment the lung parenchyma from the perspective of pathology. Dai et al. [5] used graph cut theory to extract lung parenchyma. Liao et al. [6] used the correlation of image sequences to segment lung parenchyma. Dong et al. [7] extracted lung parenchyma by regional growth method. Skourt et al. [8] constructed a deep learning network to segment lung parenchyma. Xiao et al. [9] constructed a morphological model to segment the lung parenchyma. Lv and Sun [10] improved the extraction of lung parenchyma by U-Net. Liu and Wei [11] segmented lung parenchyma based on matrix grey incident. Maity et al. [12] established CNN network to segment lung parenchyma.

*Lung nodule extraction*: Sivakumar and Chandrasekar [13] extracted lung nodules by unsupervised clustering models. Farag et al. [14] constructed level sets to segment lung nodules. Badura and Pietka [15] used 3D model to segment lung nodules. Qiang et al. [16] used the active contour model to extract the region of lung nodules. Nithila and Kumar [17] proposed active contour model and fuzzy C-mean clustering to realize lung nodule segmentation. Mukherjee et al. [18] used deep learned prior based graph cut to segment lung nodules. Liu et al. [19] constructed mask R-CNN to segment lung nodules. Aresta et al. [20] constructed an artificial interactive method to extract lung nodules. Cao et al. [21] constructed dual-branch residual network to segment lung nodules. Savic et al. [22] proposed a region-based fast marching method to achieve lung nodule segmentation. Shariaty et al. [23] constructed a model to segment lung nodules from the perspective of texture features.

*Lung nodule recognition*: Orozco et al. [24] used SVM to classify the signs of lung nodules. Zhang et al. [25] proposed multilevel patch-based context analysis for lung nodule recognition. Al et al. [26] used wavelet transform to analyze the signs of lung nodules. Shen et al. [27] constructed multiscale revolutionary neural networks to classify lung nodules. Bobadilla and Pedrini [28] used deep revolutionary neural networks to classify lung nodules. Froz et al. [29] used texture features to classify lung nodules. Wei et al. [30] established local kernel region models with out-of-sample extension to classify lung nodules. Al-Shabi et al. [31] established deep local global networks to classify lung nodules. Lei et al. [32] focused on the boundary of lung nodules to realize the classification of lung nodules under the condition of low-dose CT. Calheiros et al. [33] classified the signs of lung nodules from the surrounding conditions of lung nodules. Halder et al. [34] constructed an adaptive morphology-aided 2-path progressive neural network to segment lung nodules.

Methods of computer-aided diagnosis have been proved that they can effectively assist doctors to make accurate diagnosis. However, it is still difficult to study weak lung nodules and complex and diverse signs of lung nodules. Specifically, it includes the following: (1) the model established by the computer does not conform to the doctors' diagnosis process. (2) In the face of lung nodules with lung wall adhesion, incomplete extraction will occur and result in missed detection. (3) In the face of complex and diverse signs of lung nodules, it is impossible to accurately distinguish from a single body position.

Therefore, a new lung nodule segmentation and recognition algorithm is proposed. (1) According to the doctor's diagnosis process, a lung nodule segmentation and recognition algorithm process is constructed in line with the doctor's diagnosis process. (2) The attention mechanism is constructed to focus on the area where the lung parenchyma is located, accurately extract the lung parenchyma, and reduce the missed detection rate of lung nodules. (3) The multiposition feature enhancement network is constructed to recognize the signs of lung nodules.

## 2. Details of Algorithm

According to the diagnosis process of lung nodules by doctors, the algorithm flow is proposed, as shown in Figure 1. Firstly, the lung parenchyma extraction model of attention mechanism is established, and then, the multiposition bidirectional enhancement feature pyramid network is established to extract lung nodules. Finally, the signs of lung nodules are identified by radiomics and morphological features.

### 2.1. U-Net Algorithm

U-Net is proposed based on a fully convolutional neural network and has achieved certain results in image segmentation. U-Net consists of an encoder part and a decoder part, as shown in Figure 2. The encoder has four submodules, which are composed of a convolution layer and a pooling layer, so that the image features are gradually reduced and abstracted; the decoder corresponds to it layer by layer, and the function of the deconvolution layer in the decoder is to increase the feature size in turn and use skip connections to connect and merge the deconvolution result of the decoding part and the output of the encoding part correspondingly. Finally, the probability map is output through convolution.

In the lung parenchyma segmentation algorithm, we introduce an attention mechanism to make U-Net focus on the region of interest. And we introduced dense atrous convolution to adjust the receptive field. In the lung nodule extraction algorithm, we introduce a multiangle model into a unified U-Net to achieve multiangle detection.

### 2.2. Lung Parenchyma Segmentation Algorithm

Lung nodules only exist in the lung parenchyma. In order to simulate the diagnosis process of doctors, it is necessary to focus on the area where the lung nodules are located to realize the segmentation of lung parenchyma. It consists of encoding path and decoding path.

The traditional encoding and decoding method is U-Net, which can obtain spatial information in shallow network, but the learning ability of depth feature is not good. The cascade method leads to high redundancy in the utilization of shallow features in feature fusion, which makes the network huge. Therefore, we introduce the attention mechanism into the network to obtain higher-level features and increase the weight of the target region in order to avoid the interference of background pixels and improve the learning ability of the model.

The corresponding attention model is shown in Figure 3. The module contains two inputs, upsampling feature *g* and coding feature *x*^*l*^. Through the convolution operation of (1,1,1), *W*_*g*_^*T*^*g*_*i*_ and *W*_*x*_^*T*^*x*_*i*_^*l*^ are obtained. On this basis, an attention model is built as follows:

(1) $$\begin{array}{c} J=\sigma_{2}\left[\varphi^{T}\left(\sigma_{1}\left(W_{x}^{T}x_{i}^{l}+W_{g}^{T}g_{i}+b_{g}\right)\right)+\frac{1}{1+\exp\left(-x_{i}\right)}\right], \end{array}$$

where *φ* represents the convolution kernel.

In view of the limitations of U-Net network, the continuous pooling kernel convolution step operation reduces the resolution, which results in the loss of detail information, and increases the receptive field by expanding the convolution kernel, which results in the increase of parameters and the difficulty of training. Thus, we add a dense connected block (DAC) to improve the network and integrate inception, residual network, and hole convolution. Its structure is shown in Figure 4. Four cascade branches are used, and the corresponding receptive fields are 3, 7, 9, and 19. It is activated by ReLu. Based on the idea of residual network, the original features and other features are fused to enhance feature mining. Finally, combined with the cavity convolution of different scale expansion rates, the multiscale feature extraction is realized.

In the standard U-Net framework, the sampling function of the maximum pooling kernel is used to reduce and mediate the resolution of the feature image, respectively, but the training process will lead to feature loss and accuracy reduction. Therefore, we construct the following structure, as shown in Figure 5. The transposed convolution is to transpose the convolution kernel in the ordinary convolution operation which we usually use and then take the output of the ordinary convolution as the input of the transposed convolution, and the output of the transposed convolution is the ordinary convolution input. This structure is composed of multiscale convolution cores in parallel, which can catch up with the characteristics of different dimensions and provide the learning ability of the network.

Since lung parenchyma segmentation belongs to pixel segmentation and can be regarded as a binary classification problem, we introduce the Dice loss function to define the loss function:

(2) $$\begin{array}{c} \text{Loss}=1-\frac{2\sum_{i}^{N}p_{i}g_{i}}{\sum_{i}^{N}p_{i}^{2}+\sum_{i}^{N}g_{i}^{2}}, \end{array}$$

where *N* represents the number of pixels and *g*_*i*_ ∈ {0, 1} is used to distinguish between foreground and background. *p*_*i*_ ∈ (0, 1) represents the prediction result of the *i*-th pixel.

### 2.3. Lung Nodule Extraction and Sign Recognition Algorithm

Lung nodules have 3D features, so it is difficult to extract lung nodules from axial position alone. Therefore, we construct sagittal and coronal images according to axial images, improve U-Net network, and combine with bidirectional enhanced feature fusion network to enhance the extraction of lung nodules at different scales. The Mish activation function is introduced to shorten the network transmission time and improve the efficiency, as shown Figure 6.

The depth of the network is 5 layers, and the edge padding operation is used to replace the traditional U-Net crop operation, so that the output image size of the network is consistent with the input to realize feature fusion.

Because the high-level features mainly contain rich semantic information of the target, the low-level features mainly contain accurate location information of the target. Therefore, we build a two-way enhanced feature pyramid network to fuse the accurate low-level information with the high-level information through bottom-up path enhancement, so as to shorten the distance of information transmission.

Through two-way cross-scale connection, the low-level features of lung nodules are made full use and extracted, and the low-level fine-grained features with the high-level semantic features are better integrated. Feature vectors are enriched, the whole feature level is enhanced, and the utilization of features at all levels by the backbone network is improved. The network can also effectively extract the features of small nodules, so the problem of small target nodule loss is solved in the process of lung nodule segmentation.

Activation function is a way to introduce “nonlinearity” into neural network, which plays an important role in network training and evaluation. Liu et al. [19] proposed a new deep learning activation function, Mish activation function, which is a nonmonotonic, smooth, and continuous neural network activation function, and its function expression is as follows:

(3) $$\begin{array}{c} f\left(x\right)=x\tanh\left(\ln\left(1+e^{x}\right)\right). \end{array}$$

Mish function retains a small amount of negative information, which can allow a small negative gradient to flow in, so the information flow is ensured and the gradient disappearance problem of ReLU function in the process of back propagation is eliminated.

The size of lung nodules is not regularly the same, but the lung nodules are spherical in space and are round-like in axial, coronal, and sagittal positions. In this case, we normalized the image to 200 × 200 and extract radiomics and morphological features.

Spiculation sign is the main malignant sign of the lung. Therefore, we divided the data into training set and test set. *t*-test and LASSO algorithm are used to screen the discriminative features in the training set of radiomics label. Radiomics feature as first-order statistics, 3D shape, 2D shape, etc. which reflect the boundary and grayscale of lung nodules used for analysis. The method of 10 times cross-validation is used for fitting, and the omics logistic regression model is established. Conventional image features and clinical data are obtained by chi-square and *t*-test, and morphological logistic regression model is established. Integrate the two and make comprehensive statistics.

Through the above algorithm, it is applied to the images of lung nodules in axial, coronal, and sagittal positions, respectively. If there is at least one azimuth image that meets the spiculation sign, it is determined that the lung nodule is the spiculation sign.

## 3. Experiments and Results Analysis

The International Early Lung Cancer Action Project database is used in the experiment [35], and 500 sets of lung CT data are collected clinically. To verify the effectiveness of the algorithm, a database was constructed, including images with lung nodules, images of lung cancer, and images with grid-like increased density, as shown in Figure 7. Professional doctors are invited to outline the lung parenchyma and lung nodule areas and mark the signs of lung nodules.

The lung CT data is 16-bit data, and the image we see is an image displayed by dynamically adjusting the window width and window level, as shown in Figure 8. In terms of algorithm design, a container of 16 should be used.

Lung nodules smaller than 5 mm are called micronodules, which are generally benign and do not require special treatment. Lung nodules of 6-8 mm are partially solid nodules, so as to detect the possibility of malignant transformation as early as possible. Therefore, we focused on 6-8 mm lung nodules. Conduct studies and expand their lung nodules to a uniform size. Since spiculation has great threat to human beings and high probability of malignancy, it becomes the focus of current research.

The algorithm builds the model from the axial, coronal, and sagittal views and uses the circularity to preliminarily screen the region of interest through the segmentation algorithm to obtain the lung nodule region.

Md, Vd, Ud, and CM are introduced to measure the segmentation performance of the algorithm.

(4) $$\begin{array}{c} \text{Md}=\frac{E_{g}\cap E_{s}}{E_{g}\cup E_{s}}\times 100\%, \end{array}$$

(5) $$\begin{array}{c} \text{Vd}=\frac{E_{s}\wedge E_{g}}{E_{s}}\times 100\%, \end{array}$$

(6) $$\begin{array}{c} \text{Ud}=\frac{E_{g}\wedge E_{s}}{E_{g}}\times 100\%, \end{array}$$

(7) $$\begin{array}{c} \text{CM}=\frac{1}{3}\left\{Md+\left(1-Nd\right)+\left(1-Ud\right)\right\}\times 100\%, \end{array}$$

where *E*_*g*_ is the area outlined by the doctor, *E*_*s*_ is the area extracted by the algorithm, and ∧ represents XOR operation. Md and CM are directly proportional to the algorithm performance, and Vd and Ud are inversely proportional to the algorithm performance.

SEN, SPE, FPF, and ROC are introduced to measure the recognition performance:

(8) $$\begin{array}{c} \text{SEN}=\frac{\text{TP}}{\text{TP}+\text{FN}}, \end{array}$$

(9) $$\begin{array}{c} \text{SPE}=\frac{\text{TN}}{\text{TN}+\text{FP}}, \end{array}$$

(10) $$\begin{array}{c} \text{FPF}=\frac{\text{FP}+\text{FN}}{\text{TP}+\text{FP}+\text{TN}+\text{FN}}. \end{array}$$

### 3.1. Performance of Lung Parenchyma Segmentation Algorithm

The performance of the algorithm is shown in Table 1. Reference [4] builds a 3D model to realize extraction of lung parenchyma. Reference [5] used graph cuts to build an energy model to guide lung parenchyma segmentation. Reference [10] constructed U-Net from the perspective of deep learning to extract lung parenchyma pairs and achieved certain positive results. The above algorithm is not effective for the extraction of lung nodules and lung parenchyma with lung wall adhesions that are relatively close. However, this paper proposes an algorithm to build an attention mechanism, reduces the amount of parameters, focuses on the lung parenchyma area, and realizes the extraction of lung parenchyma. The effect is shown in Figure 9, and good results are achieved.

### 3.2. Performance of Lung Nodule Segmentation Algorithm

The algorithm performance is shown in Table 2. Level set algorithm [14] focuses on the boundary of lung nodules and extracts lung nodules. Active contour model [16] extracts lung nodules. Dual-branch residual network [21] realizes lung nodule segmentation. The extraction effect of the algorithm proposed is shown in Figure 10. It can be seen that the algorithm constructs a bidirectional enhanced feature pyramid network from three body positions to realize lung nodule segmentation, and the effect is better than other algorithms.

### 3.3. Performance of Lung Nodule Sign Recognition Algorithm

We constructed axial, coronal, and sagittal models to judge the characteristics of lung nodules from three positions. Lung nodule recognition result is show in Table 3. It has high detectability for isolated lung nodules, and the detection rate of lung nodules with vascular adhesion is slightly low, but the overall trend is upward.

The lung nodules are spherical, and the lung nodules cannot be accurately targeted from only one position, so they are reflected from multiple positions. In the nodular region as shown in Figure 11(a), it will appear as a circle in a single position, and it may appear as a long strip from other positions as show in Figure 11(b), which can be judged as a nonlung nodule region. In turn, then the advantages of the multiposition algorithm are reflected.

The performance of the algorithm is shown in Table 4, and its ROC curve is shown in Figure 12. Ref [29] extracted texture features to classify lung nodules. Ref [27] constructed multiscale revolutionary neural networks to recognize the signs of lung nodules. The proposed algorithm realizes the signs of lung nodules by texture information and image radiomics features and has a good effect.

## 4. Conclusion

Aiming at the difficult problem of lung nodule segmentation and sign recognition, we constructed a lung nodule segmentation and recognition algorithm based on multiposition U-Net from the doctor's diagnosis process. From the perspective of lung parenchyma segmentation, lung nodule segmentation, and lung nodule recognition, the attention mechanism model, multiposition feature enhancement model, morphology, and radiomics model are constructed, respectively, and finally, the automatic recognition of lung nodule signs can be realized, which can assist doctors to make accurate diagnosis.

## Figures and Tables

**Figure 1:** Algorithm flow chart.

**Figure 2:** U-Net.

**Figure 3:** Internal structure of attention mechanism.

**Figure 4:** Dense atrous convolution block.

**Figure 5:** Sampling structure.

**Figure 6:** Network structure.

**Figure 7:** Database display.

**Figure 8:** Image of different window width and window level.

**Figure 9:** Effect graphs of lung parenchyma segmentation.

**Figure 10:** Segmentation effect of lung nodules.

**Figure 11:** Nodule and vessel images.

**Figure 12:** ROC.

**Table 1:** Comparison of lung parenchyma segmentation performance.

Algorithm	Md (%)	Vd (%)	Ud (%)	CM (%)
3D	86	13	14	86
Graph cuts	87	12	16	86
U-Net	95	10	13	90
Ours	98	8	10	93

**Table 2:** Comparison of segmentation performance of lung nodules.

Algorithm	Md (%)	Vd (%)	Ud (%)	CM (%)
Level sets	79	21	20	79
Active contour model	83	20	18	81
Dual-branch residual network	86	17	15	84
Ours	91	15	11	88

**Table 3:** Lung nodule recognition rate.

FPF (%)	Axial	Axial+coronal	Axial+coronal+sagittal
Isolated nodules	89	93	95
Vascular adhesive nodule	78	85	91

**Table 4:** Performance comparison of feature recognition algorithms.

Algorithm	SEN (%)	SPE (%)	FPF (%)
Texture	79	74	20
SVM	81	79	19
MSCN	84	83	18
Ours	91	88	15

## Data Availability

The International Early Lung Cancer Action Project can be accessed through the link (https://veet.via.cornell.edu/lungdb.html). For the clinical data used to support the findings of this study, they are available from the corresponding author upon request.
